# Efficacy of Low Molecular Heparin on Preeclampsia by Inhibiting Apoptosis of Trophoblasts via the p38MAPK Signaling Pathway

**DOI:** 10.1155/2021/3337514

**Published:** 2021-08-02

**Authors:** Dandan Quan, Li Li, Manzhen Zuo

**Affiliations:** ^1^Department of Obstetrics and Gynecology, The People's Hospital of China Three Gorges University, The First Hospital of Yichang, Hubei 443000, China; ^2^Department of Obstetrics and Gynecology, The Affiliated Jiangning Hospital of Nanjing Medical University, Nanjing 211100, China

## Abstract

**Objective:**

To explore the efficacy of low molecular heparin on preeclampsia by inhibiting apoptosis of trophoblasts via the p38MAPK signaling pathway.

**Methods:**

A preeclampsia rat model was established, and the effects of low molecular heparin on preeclampsia via the p38MAPK signaling pathway were analyzed based on intervention of the rats with different combinations of low molecular heparin and p38MAPK signaling pathway activator. Furthermore, a hypoxia/reoxygenation model of trophoblasts in vitro was established to explore the effects of low molecular heparin on trophoblasts via the p38MAPK signaling pathway.

**Results:**

After treatment with low molecular heparin, pregnant rats in the heparin group showed significantly decreased blood pressure, 24 h proteinuria, and p38MAPK protein levels in placenta tissues and decreased apoptosis rate of placenta tissue cells (all *P* < 0.05) and showed more fetal rats and lowered weight of them (both *P* < 0.05) but showed no significant change in the weight of placenta (all *P* > 0.05). Pregnant rats treated with low molecular heparin and p38MAPK activator showed significantly higher blood pressure, 24 h proteinuria, and p38MAPK protein levels in placenta tissues and apoptosis rate of placenta tissue cells than those of pregnant rats in the heparin group (all *P* < 0.05) and also showed less fetal rats and lighter fetal rats than those in the heparin group (both *P* < 0.05) but showed no difference with them in the weight of placenta (*P* > 0.05). Further analysis revealed that low molecular heparin could protect the survival and migration of trophoblasts under hypoxia/reoxygenation conditions and reduce apoptosis of them (all *P* < 0.05).

**Conclusion:**

Low molecular heparin can alleviate preeclampsia by inhibiting the p38MAPK signaling pathway and can inhibit apoptosis of trophoblasts and promote proliferation and migration of them.

## 1. Introduction

Preeclampsia is a leading cause of premature delivery of infants and maternal and infant mortality. Its clinical manifestations include hypertension and placenta, and its incidence is about 2%-5% [1]. At present, some scholars believe that preeclampsia is correlated with maternal childbearing age and placenta, and it is generally believed that preeclampsia is caused by reperfusion injury after placental ischemia, oxidative stress, and imbalance of angiogenesis/antiangiogenic factors, and it is prone to cause lifelong complications of cardiovascular and kidney diseases in women, increasing the risk of stroke in women by 6 times [2, 3].

Low molecular heparin is often used to prevent preeclampsia, which can lower the occurrence of preeclampsia and reduce fetal death [4, 5]. However, as many researches only focus on the analysis of the efficacy of low molecular heparin, the mechanism of it in preventing preeclampsia has not been fully studied. Trophoblasts are the main cellular form of placenta, with an important role in the development and progression of preeclampsia [6]. Some studies have reported that low molecular heparin can protect trophoblasts and maintain their functions [7, 8]. Interestingly, the p38MAPK signaling pathway has effects similar to those of low molecular heparin [9, 10], which suggests that low molecular heparin may affect preeclampsia like the p38MAPK signaling pathway. It has been reported that activating the MAPK signaling pathway is an action mechanism of low molecular heparin in promoting the migration of trophoblasts [11].

This study has analyzed the effects of low molecular heparin on trophoblasts to explore its therapeutic mechanism.

## 2. Materials and Methods

### 2.1. Research Objects

Sixty specific pathogen-free (SPF) Wistar rats were purchased from the Animal Center of Southern Medical University, with animal license of SCXK (Yue) 2016-0041, including 30 female rats between 8 and 10 weeks old, with weight of 200-220 g and 30 male rats between 9 and 11 weeks old, with weight of 300-330 g. The rats were raised in 30 cages with one male rat and one female rat in each cage at room temperature of 20-25°C under relative humidity of 40%-70% and a light/dark cycle of 12 hours, and they were allowed to freely drink water. Then, the vaginal suppository of each female rat was analyzed on the next day. All animal experiments were carried out under the approval by the Animal Care and Use Committee of our hospital and the guiding principles of the Council for International Organization of Medical Sciences (CIOMS).

### 2.2. Establishment of Preeclampsia Model

On the 13^th^ day after the formation of vaginal suppository in female rats, the blood pressure of each female rat was measured and recorded. Then, 30 female rats were selected by the random number table method, and each selected female rat was subcutaneously injected with 200 mg/(kg·d) L-nitroarginine methyl ester (Sigma Company, the United States) for 4 consecutive days. If the blood pressure of a selected rat increased by more than 30 mmHg, the modeling of the rat was considered successful. The used animal sphygmomanometer was purchased from Shanghai Yuyan Scientific Instruments Co., Ltd.

### 2.3. Grouping and Treatment of Rats

Twenty-four of the 30 female rats were successfully modeled, and they were assigned to a model group, a low molecular heparin intervention group (hereinafter referred to as the heparin group), and a low molecular heparin combined with p38MAPK activator intervention group (hereinafter referred to as the combination group), 8 rats in each group. The rest 10 female rats were taken as a control group. Female rats in the heparin group were injected intravenously with 40 *μ*L/(kg d) low molecular heparin at the 15^th^ day after vaginal suppository was formed, and rats in the combination group were injected intravenously with 0.5 mg/kg p38MAPK activator through tail vein on the basis of treatment to those in the heparin group. Rats in the control group and the model group were injected subcutaneously with the same volume of normal saline as that of low molecular heparin. On the 21^st^ day after pregnancy of each rat, the pregnant rat was anesthetized with 3% pentobarbital sodium by intraperitoneal injection to take the fetal rats and placenta out, and the number of fetal rats and weight of them and apoptosis rate of placenta tissue cells were recorded. The low molecular heparin was purchased from GlaxoSmithKline (Tianjing, China), and the p38MAPK activator (Dehydrocorydaline chloride) was from the MCE Company in China. In addition, pentobarbital sodium was purchased from Shanghai Kefeng Chemical Reagent Co., Ltd., and electronic scales from Beijing Jinda Sunshine Technology Co., Ltd.

### 2.4. Blood Pressure and Proteinuria Detection

The blood pressure and 24 h proteinuria of pregnant rats were recorded before modeling, after 15 days of pregnancy, and 21 days of pregnancy, respectively, and the 24 h proteinuria was analyzed using an automatic biochemistry analyzer (SYSMEX BX-4000 full-automatic biochemical analyzer) from SYSMEX Medical Electronics (Shanghai) Co., Ltd.

### 2.5. Detection of p38MAPK Signaling Pathway-Related Proteins

A Western blot assay was carried out to detect the p38MAPK level, and the protein of tissues and cells was extracted using the freeze-thaw method. The concentration of the protein was determined using the bicinchoninic acid (BCA) method and adjusted to 4 *μ*g/*μ*L. The protein was separated through 12% polyacrylamide gel electrophoresis. The initial voltage was 90 V, and then, the voltage was increased to 120 V to move the sample to an appropriate position of the separation gel. After electrophoresis, the protein was transferred to a membrane under 100 V constant voltage for 100 min and blocked at 37°C for 60 min. Subsequently, the membrane was blocked with 5% skim milk powder for future immune response. The membrane was incubated with primary antibody (1 : 1000) at 4°C for one night and then washed with warm phosphate buffer saline (PBS) three times, 5 min each time. After washing, the membrane was incubated with secondary antibody (1: 1000) at room temperature for 1 h. After incubation, the protein was developed and immobilized with electrochemiluminescence (ECL) agent. The scanned protein band was analyzed using the Quantity One software, and the relative protein expression level was recorded as the gray value of the band/gray value reference. BCA protein kit, ECL kit, and trypsin with item numbers of 23250, 35055, and 90058 were all purchased from Thermo Scientific™, and rabbit anti-p38MAPK, bcl-2, bax monoclonal antibodies, and goat anti-rabbit IgG secondary antibodies with item numbers of ab170099, ab185002, ab32503, and ab6721 were all purchased from the Abcam Company in the United States.

### 2.6. Cell Apoptosis Experiment by the Tunel Method

The apoptosis rates of placenta tissue cells and chorionic villus cells were measured using the Tunel method as follows: The number of apoptotic cells and the total number of cells under five selected fields under an optical microscope were counted, and the apoptosis rate was calculated.

### 2.7. Cell Sources

Human chorionic villus cells (HTR-8/Svneo) with number of CRL-3271 purchased from the American Type Culture Collection (ATCC) were cultured in RPMI-1640 medium with 5% fetal bovine serum in 95% air and 5% carbon dioxide at 37°C.

### 2.8. Cell Grouping and Intervention

The cells were assigned into a blank group, a hypoxia group, a heparin group, and a combination group. Except for cells in the blank group, cells in other groups were all treated with hypoxia/reoxygenation (hypoxia for 2 hours and reoxygenation for 4 hours). Cells in the heparin group in medium were added with 5% heparin, and cells in the combination group were added with 5% heparin and 5% p38MAPK activator. Afterwards, the apoptosis and migration of the cells were detected.

### 2.9. Cell Proliferation Assay by Cell Counting Kit-8 (CCK8)

A total of 1∗10^3^ cells were routinely seeded into a 96-well plate, and 10 *μ*L CCK8 solution was added into the cells at 24 h, 48 h, 72 h, and 96 h after culturing, respectively. The optical density of each well at 450 nm was measured using a microplate reader (Bio Rad, Hercules, California, the United States) after each addition of CCK8 solution.

### 2.10. Determination of Migration and Invasion of Cells

A total of 5 × 10^4^ cells were transferred to the upper compartment, and the lower compartment was added with L-15 medium with 10% FBS. Twenty-four hours later, the cells under the microporous membrane were immobilized with 75% methanol and stained with crystal violet. Subsequently, the number of cells penetrating the membrane in five selected fields under an optical microscope was calculated, and three parallel experiments were carried out. The Transwell insert and related reagents were purchased from Corning (New York, the United States).

### 2.11. Statistical Analysis

In this study, the data were statistically analyzed and visualized into figures using Graphpad Prism 8, and measurement data were expressed as the mean ± standard deviation. Comparison among multiple groups was conducted using the one-way ANOVA, and back testing was carried out using LSD. In addition, Pearson's analysis was used for correlation analysis. *P* < 0.05 indicated a significant difference.

## 3. Results

### 3.1. Efficacy of Different Interventions on Preeclampsia in Pregnant Rats

Compared with pregnant rats in the control group, pregnant rats in the model group showed significantly higher blood pressure and 24 h proteinuria levels (both *P* < 0.05) and showed significantly less fetal rats, lighter fetal rats, and placenta (all *P* < 0.05), suggesting that the modeling was successful. In addition, after treatment with low molecular heparin, pregnant rats in the heparin group showed significantly decreased blood pressure and 24 h proteinuria levels (both *P* < 0.05) and showed an increase in the number of fetal rats and weight of them but showed no significant change in the weight of placenta (*P* > 0.05). Rats in the combination group showed significantly higher blood pressure and 24 h proteinuria, less fetal rats, and lighter fetal rats than those in the heparin group (all *P* < 0.05) but showed no difference with them in the weight of placenta (*P* > 0.05) (Figure 1).

### 3.2. Effects of Different Interventions on the p38MAPK Protein Level in Placenta Tissues of Pregnant Rats

The p38MAPK protein level in placenta tissues was seen in the model group, the combination group, the heparin group, and the control group from high to low (all *P* < 0.05) (Figure 2).

### 3.3. Effects of Different Interventions on Apoptosis of Placenta Tissue Cells of Pregnant Rats

The apoptosis of placenta tissue cells and the level of apoptosis-related protein (bax) were both seen in the model group, the combination group, the heparin group, and the control group from high to low (all *P* < 0.05), and the level of apoptosis-related protein (bcl-2) was seen in them from low to high (all *P* < 0.05). Correlation analysis showed that the level of p38MAPK protein was significantly linearly correlated with the apoptosis rate, bax, and bcl-2 levels of placenta tissue cells (all *P* < 0.05) (Figure 3).

### 3.4. Effects of Different Interventions on the p38MAPK Protein Level in Chorionic Villus Cells

The level of p38MAPK protein in chorionic villus cells was seen in the blank group, the heparin group, the combination group, and the hypoxia group from low to high (all *P* < 0.05) (Figure 4).

### 3.5. Effects of Different Interventions on Apoptosis of Chorionic Villus Cells

The apoptosis rate of chorionic villus cells and the level of apoptosis-related protein (bax) were both seen in the hypoxia group, the combination group, the heparin group, and the control group from high to low (all *P* < 0.05), and the level of apoptosis-related protein (bcl-2) was seen in them from low to high (all *P* < 0.05) (Figure 5).

### 3.6. Effects of Different Interventions on Proliferation and Migration of Chorionic Villus Cells

The proliferation and migration abilities of chorionic villus cells were seen in the hypoxia group, the combination group, the heparin group, and the control group from low to high (all *P* < 0.05) (Figure 6).

## 4. Discussion

Preeclampsia is the major cause of perinatal morbidity and mortality for pregnant and lying-in women all over the world. Excessive death of placental cells is a crucial clinical manifestation of women with preeclampsia, which leads to maternal placental dysfunction and induces thrombosis, abortion, etc. [12, 13]. Low molecular heparin can improve the placental function by increasing blood flow to the implantation site and reduce the thrombosis [14]. Studies show that low molecular heparin can promote the angiogenesis and suppress apoptosis of trophoblasts [15, 16]. However, the mechanism of this action of low molecular heparin remains unclear. This study found that low molecular heparin could suppress the apoptosis of trophoblasts and could promote proliferation and migration of them by inhibiting the p38MAPK signaling pathway.

In this study, we constructed preeclampsia rat models through L-nitroarginine methyl ester [17], finding that blood pressure and 24 h proteinuria levels of the rats significantly increased and the number of fetal rats and weight of them and the weight of placenta in them decreased significantly. In addition, we also found that the apoptosis rate of placenta tissue cells of the rats increased significantly, while after intervention of low molecular heparin, those manifestations were improved. The results were consistent with previous research results. Low molecular heparin can positively act on preeclampsia [18, 19]. The p38MAPK signaling pathway has been reported to be related to the growth and migration of trophoblasts. For example, a study by Zhou et al. [20] has revealed that transforming growth factor-*β*1 could inhibit the apoptosis of trophoblasts induced by mercuric chlorides by suppressing the p38MAPK signaling pathway, and one other study by Ebegboni et al. [21] also reported that flavonoids promoted the self-renewal and invasion of spherical stem cells of trophoblasts by inhibiting p38MAPK signaling pathway. In addition, one study by Che et al. [22] also found that knockout of heparanase gene inhibits the invasion of human trophoblasts by activating the p38MAPK signaling pathway. Heparin has also been reported to inhibit excessive circulation and remodeling of porcine pulmonary artery via the p38MAPK signaling pathway, thus alleviating the pulmonary hypertension [23]. Low molecular heparin, as a derivative of heparin, may also play its role by regulating the p38MAPK signaling pathway, but no research on it has been reported so far. In this study, we found that low molecular heparin could inhibit the p38MAPK signaling pathway. According to the design idea of rescue experiment, we activated the p38MAPK signaling pathway under the intervention with low molecular heparin, finding that the efficacy of low molecular heparin was strongly inhibited and the apoptosis of placental tissue cells was also significantly lowered. Therefore, we can conclude that low molecular heparin could alleviate preeclampsia by inhibiting the p38MAPK signaling pathway and could lower the apoptosis of placenta tissue cells. In order to further verify the effects of low molecular heparin on trophoblasts via the p38MAPK signaling pathway, we used an in vitro hypoxia-reoxygenation model to simulate the living environment of trophoblasts in preeclampsia patients, finding that low molecular heparin could protect trophoblasts via the p38MAPK signaling pathway.

There are some deficiencies in this study. For example, the effects of low molecular heparin on inhibiting the p38MAPK signaling pathway have been verified only in rats, but the onset of preeclampsia is complicated, such as significant differences in the condition and prognosis between patients with early-onset preeclampsia and those with late-onset preeclampsia. In addition, one study by Bolnick et al. [7] has uncovered that low molecular heparin induces extracellular differentiation of trophoblasts through epidermal growth factor-like growth factor signals and reduces apoptosis of them during oxidative stress, which indicates that there are more mechanisms for the influence of low molecular heparin on trophoblasts, so a large amount of research is needed for exploration of the mechanisms.

To sum up, low molecular heparin can alleviate preeclampsia by inhibiting the p38MAPK signaling pathway and can inhibit apoptosis of trophoblasts and promote proliferation and migration of them.

## Figures and Tables

**Figure 1:** Efficacy of different interventions on preeclampsia in pregnant rats. (a) Blood pressure; (b) 24 h proteinuria; (c) the number of fetal rats; (d) the weight of fetal rats; (e) the weight of placenta. a indicates that in comparison with the control group, *P* < 0.05; b indicates that in comparison with the model group, *P* < 0.05, and c indicates that in comparison with the heparin group, *P* < 0.05.

**Figure 2:** Effects of different interventions on the p38MAPK protein level in placenta tissues of pregnant rats. a indicates that in comparison with the control group, *P* < 0.05; b indicates that in comparison with the model group, *P* < 0.05, and c indicates that in comparison with the heparin group, *P* < 0.05.

**Figure 3:** Effects of different interventions on apoptosis of placenta tissue cells of pregnant rats. (a) Apoptosis rate of placenta tissue cells; (b) the bax protein level in placenta tissues; (c) the bcl-2 protein level in placenta tissues; (d) the correlation between p38MAPK protein level and apoptosis rate in placenta tissue cells; (e) the correlation between p38MAPK and bcl-2 protein level in placenta tissues; (f) the correlation between p38MAPK and bax protein level in placenta tissues. a indicates that in comparison with the control group, *P* < 0.05; b indicates that in comparison with the model group, *P* < 0.05, and c indicates that in comparison with the heparin group, *P* < 0.05.

**Figure 4:** Effects of different interventions on the p38MAPK protein level in chorionic villus cells. a indicates that in comparison with the control group, *P* < 0.05; b indicates that in comparison with the hypoxia group, *P* < 0.05, and c indicates that in comparison with the heparin group, *P* < 0.05.

**Figure 5:** Effects of different interventions on apoptosis of chorionic villus cells. (a) Apoptosis rate of chorionic villus cells; (b) bax protein level in chorionic villus cells; (c) bcl-2 protein level in chorionic villus cells. a indicates that in comparison with the control group, *P* < 0.05; b indicates that in comparison with the hypoxia group, *P* < 0.05, and c indicates that in comparison with the heparin group, *P* < 0.05.

**Figure 6:** Effects of different interventions on proliferation and migration of chorionic villus cells. (a) Analysis of proliferation ability of chorionic villus cells; (b) analysis of migration ability of chorionic villus cells. a indicates that in comparison with the control group, *P* < 0.05; b indicates that in comparison with the hypoxia group, *P* < 0.05, and c indicates that in comparison with the heparin group, *P* < 0.05.

## Data Availability

All the raw data could be accessed by contacting the corresponding author if any qualified researcher need.
